# Relationship between Admission Electrolyte Level and Short-term Prognosis of Patients with Acute ST-segment Elevation Myocardial Infarction after Percutaneous Coronary Intervention

This article has been retracted.

**DOI:** 10.1155/2021/4664965

**Published:** 2021-08-09

**Authors:** Yaping Ren, Zhijie Yue, Xuewen Li

**Affiliations:** ^1^Department of Internal Medicine-Cardiovascular, Shanxi Bethune Hospital, Shanxi Academy of Medical Sciences, Tongji Shanxi Hospital, Third Hospital of Shanxi Medical University, Taiyuan 030032, Shanxi, China; ^2^Department of Internal Medicine-Cardiovascular, Tongji Hospital, Tongji Medical College, Huazhong University of Science and Technology, Wuhan 430030, Hubei, China

## Abstract

**Objective:**

The objective of this study is to analyze the relationship between the electrolyte level of patients with acute ST-segment elevation myocardial infarction (STEMI) and short-term prognosis after percutaneous coronary intervention (PCI).

**Methods:**

The clinical data of 142 patients with acute STEMI who underwent PCI in our hospital from September 2018 to September 2019 were retrospectively analyzed. According to the level of serum sodium, potassium, and chloride in patients admitted to the hospital, they were divided into the normal electrolyte group (*n* = 78), the mild decline group (*n* = 46), and the severe decline group (*n* = 16). Univariate and logistic regression multivariate analysis of the relationship between patient electrolyte levels and general clinical data is performed. Statistical analysis of patients' adverse events within 90 days was performed. The Kaplan–Meier survival curve analyzed the relationship between the survival period and electrolyte levels in patients with acute STEMI without major acute cardiovascular events (MACE) within 90 days.

**Results:**

The levels of creatine kinase-MB (CK-MB), cardiac troponin I (cTnI), myocardial infarction area, and Gensini score in patients with mild decline were significantly higher than those in the normal group, left ventricle ejection fractions (LVEF) value was significantly lower than the normal group, and patients with severe decline were significantly higher in creatine kinase (CK) level than the normal group (*P* < 0.05). The levels of CK-MB, CK, cTnI, and myocardial infarction area of the patients in the severe decline group were significantly higher than those in the mild decline group, and the LVEF values were significantly lower than those in the mild decline group (*P* < 0.05). The levels of CK-MB, CK, cTnI, the area of myocardial infarction, and Gensini score in patients with acute STEMI have an independent effect on their electrolyte levels. The patients in the mild decline group and severe decline group had significantly higher rates of cardiogenic shock, heart failure, ventricular aneurysm formation, ventricular septal perforation, or death within 90 days after PCI. The median without MACE survival time of patients with mildly and severely reduced electrolyte levels was significantly lower than that of patients with normal electrolyte levels.

**Conclusion:**

Patients with acute STEMI are prone to electrolyte disturbances, and their CK-MB, CK, and cTnI levels; myocardial infarction area; and Gensini score have independent effects on electrolyte levels. Patients with electrolyte disturbances are prone to poor prognosis after PCI, and their survival period without MACE at 90 days is significantly lower than that of normal patients.

## 1. Introduction

Acute ST-segment elevation myocardial infarction (STEMI) is the formation of occlusive thrombi on the basis of coronary atherosclerotic plaque lesions, resulting in continuous or complete obstruction of the coronary artery lumen and leading to myocardial injury and necrosis, cardiac insufficiency, and so on, whose ECG shows abnormal ST-segment elevation [1]. At present, the treatment of acute STEMI mainly includes thrombolytic therapy, percutaneous coronary intervention (PCI), emergency coronary artery bypass grafting (CABG), and so on. Among them, PCI, as an important method for the treatment of acute STEMI, has the advantages of less trauma and good postoperative recovery. It can effectively dredge the occluded infarcted blood vessel, realize coronary reperfusion, and restore the infarcted myocardium to the greatest extent [2, 3]. Electrolyte homeostasis plays an important role in maintaining normal cell metabolism, intracellular fluid osmotic pressure, acid–base balance, and nerve excitement. The abnormality of myocardial excitability and conductivity caused by the body's electrolyte disturbance can lead to different degrees of arrhythmia, and severe cases can cause myocardial infarction, cardiac arrest, and so on. At the onset of myocardial infarction, a series of intense stress reactions caused by myocardial ischemia and hypoxia, such as abnormal release of various hormones, can cause the body's blood sodium, blood potassium, and blood chloride levels to decrease, which further increases the chance of patient's malignant arrhythmia and heart failure [4, 5]. This study retrospectively analyzed the electrolyte levels of selected patients at admission and aimed to explore the relationship between the electrolyte levels of acute STEMI patients and the short-term prognosis after PCI to provide clinical guidance for improving the prognosis of acute STEMI patients. The specific research is as follows:

## 2. Materials and Methods

### 2.1. Research Object

The clinical data of 142 patients with acute STEMI who underwent PCI in our hospital from September 2018 to September 2019 were collected, including age, gender, history of diabetes, and history of hypertension. Among them, 74 were males and 68 were females, aged from 32 to 81 years old, with an average age of (60.45 ± 14.96) years old. Inclusion criteria are as follows: acute STEMI was diagnosed; the time from onset to hospital admission was less than 12 h; PCI treatment was accepted; clinical data were complete. Exclusion criteria are as follows: patients with chronic liver and kidney dysfunction, malignant tumors, and so on and patients with other diseases that may cause electrolyte imbalance.

### 2.2. Research Methods

All patients received peripheral venous blood on admission. The automatic biochemical analyzer is used to determine the level of routine electrolytes (including blood potassium, blood sodium, blood chlorine, etc.), white blood cell (WBC) count, red blood cell (RBC) count, hemoglobin (Hb), platelet (PLT) count, and creatine kinase Myocardial enzymes (CK-MB), creatine kinase (CK) and troponin (cTnI) levels, blood glucose and blood lipid levels. Echocardiography is used to determine left ventricular ejection fraction (LVEF), diastolic blood pressure (LVDP), and systolic blood pressure (LVSP). ECG combined with echocardiography is used to determine the area of myocardial infarction. All patients underwent coronary angiography, and their Gensini score was obtained by multiplying the lesion vascular stenosis score and the stenosis site coefficient.

According to the electrolyte results, patients were divided into the normal group (*n* = 78), the mild decline group (*n* = 46), and the severe decline group (*n* = 18). Electrolyte evaluation standard: normal, blood sodium 137∼147 mmol/L, blood potassium 3.50∼5.50 mmol/L, blood chlorine 100∼110 mmol/L; mild decrease, blood sodium 120∼136 mmol/L, blood potassium 3.00∼3.49 mmol/L, blood chlorine 90∼99 mmol/L; severe decrease, blood sodium <120 mmol/L, blood potassium <3.00 mmol/L, blood chlorine <90 mmol/L. The classification criteria are determined by the most severely decreased indexes in blood sodium, blood potassium, and blood chlorine.

After PCI, patients and their families were followed up by consulting medical records, outpatient clinics, and telephone. Cardiogenic shock, heart failure, ventricular wall formation, and ventricular septal perforation and other adverse events in patients were counted within 90 days. This study takes the occurrence of the aforementioned major adverse cardiovascular events (MACE) or death as the end point and records the time when the patients have MACE events.

### 2.3. Statistical Methods

The SPSS19.0 software was used for data processing, the measurement data were expressed as mean ± standard deviation ($\bar{x}\pm s$), and the comparison between multiple groups is analyzed using the F-test. The enumeration data were expressed by (%), and the comparison between groups was analyzed by *χ*^2^ -test. The logistic regression model was analyzed by multivariate analysis. The Kaplan-Meier survival curve was used to analyze the relationship between electrolyte levels and short-term MACE-free survival in patients with acute STEMI, and the log-rank test was used for comparison. The test level is *α* = 0.05, and *P* < 0.05 indicates that the difference is statistically significant.

## 3. Results

### 3.1. Comparison of General Data of Three Groups of Acute STEMI Patients

The analysis results showed that the levels of CK-MB and cTnI, myocardial infarction area, and Gensini score of the patients in the mild decline group and the severe decline group were significantly higher than those in the normal group, and the LVEF value was significantly lower than that in the normal group, the CK level in the severe decline group was significantly higher than that in the normal group, the difference was statistically significant (*P* < 0.05); the levels of CK-MB, CK, and cTnI; myocardial infarction area; and Gensini score of the severe decline group were significantly higher than those of the mild decline group, and the LVEF value was significantly lower than that in the mild decline group, the differences were statistically significant (*P* < 0.05). As show in Table 1.

### 3.2. Analysis of Multiple Factors Affecting Electrolyte Levels in Patients with Acute STEMI

The results of multivariate analysis showed that the levels of CK-MB, CK, and cTnI; myocardial infarction area; and Gensini score of patients with acute STEMI have independent influence on their electrolyte levels, as shown in Table 2.

### 3.3. Statistics of Adverse Conditions in Three Groups of Acute STEMI Patients within 90 days after PCI

The results showed that the incidence of cardiogenic shock, heart failure, ventricular aneurysm formation, or ventricular septal perforation in the mild decline group and the severe decline group within 90 days after PCI was significantly higher than those in the normal group (*P* < 0.05). The incidence of heart failure, ventricular aneurysm formation, or ventricular septal perforation in the severe decline group was significantly higher than those in the mild decline group within 90 days after PCI (*P* < 0.05). The death rate of the mild decline group and the severe decline group was higher than that of the normal group, and the death rate of the severe decline group was higher than that of the mild decline group (*P* < 0.05), as shown in Table 3.

### 3.4. Relationship between Electrolyte Levels and MACE-Free Survival in Patients with Acute STEMI

As of December 2019, of the 142 follow-up patients, seven were lost to follow-up and 32 died. The median MACE-free survival time of patients in the mild decline group and the severe decline group were 65 days and 52 days, respectively, which were significantly lower than the 90 days of the median MACE-free survival time of patients in the normal group. The log-rank test was *P*=0.021, *P*=0.003, the difference was statistically significant (*P* < 0.05), as shown in Figure 1.

## 4. Discussion

Electrolyte disorders are very common in patients with acute STEMI, especially blood sodium, blood potassium, and blood chloride levels are reduced [6, 7]. It is currently believed that the neuroendocrine changes in patients with acute STEMI can promote the release of catecholamines and other hormones, increase the permeability of cell membranes, and accelerate the excretion of Na^+^, K^+^, and Cl^−^, resulting in a decrease in blood sodium, blood potassium, and blood chloride levels. In addition, when acute STEMI occurs, the ion pump activity on the cell membrane is inhibited due to ischemia and hypoxia, which will also reduce the blood sodium, blood potassium, and blood chloride levels [8, 9]. The current basic principles for the treatment of acute STEMI mainly include improving blood perfusion, saving damaged myocardial tissue, reducing the area of myocardial infarction and myocardial ischemia, and protecting heart function as much as possible [10]. PCI technology can unblock the blocked blood vessels in patients with acute STEMI in time and restore the infarcted myocardium. However, owing to the disorder of the patient's body electrolyte levels, patients with acute STEMI are prone to poor prognosis after PCI [11].

The results of this study showed that the levels of CK-MB and cTnI, myocardial infarction area, and Gensini score of patients in the mild decline group and the severe decline group were significantly higher than those of the normal group, and the LVEF value was significantly lower than that of the normal group, and the CK level of patients in the severe decline group was significantly higher than that in the normal group. Acute STEMI patients' CK-MB, CK, and cTnI levels; myocardial infarction area; and Gensini score have independent influence on their electrolyte levels. After coronary artery occlusion in patients with acute STEMI, myocardial tissue has obvious ischemia-reperfusion injury, resulting in a decrease in blood sodium, blood potassium, and blood chloride levels and a rapid increase in Na^+^, K^+^, and Cl^−^ levels in the myocardium. At this time, with myocardial cells in a hypertonic environment, it causes shrinkage and necrosis of myocardial cells, promotes the release of myocardial enzymes, and aggravates myocardial damage [12]. In addition, with the increase in the area of myocardial infarction, patients will experience myocardial remodeling, abnormal systolic and diastolic functions of the myocardium, and decreased cardiac function. The decreased cardiac function can activate the patient's neuroendocrine system and further aggravate the abnormal electrolyte level; this vicious circle seriously affects the prognosis of patients [13, 14]. The higher the Gensini score, the more severe the condition of patients with acute STEMI [15]. Related studies have confirmed that the patient's admission blood sodium, potassium, and chloride levels are negatively correlated with CK-MB, CK, cTnI levels; myocardial infarction area; and Gensini score, and positively correlated with LVEF values, with the decrease of blood sodium, blood potassium, and blood chloride levels, the levels of CK-MB, CK, and cTnI increase; the area of myocardial infarction increases; the Gensini score increases; and the LVEF value decreases [16]. This coincides with the results of this research. As of December 2019, the incidence of cardiogenic shock, heart failure, ventricular aneurysm formation, or ventricular septal perforation in the mild decline group and the severe decline group within 90 days after PCI was significantly higher than those in the normal group. The incidence of heart failure, ventricular aneurysm formation, or ventricular septal perforation in the severe decline group was significantly higher than that in the mild decline group within 90 days after PCI. Among 142 follow-up patients, seven lost follow-up and 32 died. The median MACE-free survival time of patients in the mild decline group and the severe decline group were 65 days and 52 days, respectively, which were significantly lower than the 90-day median MACE-free survival time of patients in the normal group. It is suggested that blood sodium, blood potassium, and blood chlorine levels can be used as indicators for judging the prognosis of patients with acute STEMI, and the probability of death of patients increases with the decrease of blood sodium, blood potassium, and blood chlorine levels [17, 18].

## 5. Conclusion

Acute STEMI patients are prone to electrolyte disturbances, and their CK-MB, CK, cTnI levels; myocardial infarction area; Gensini score; and electrolyte levels have independent effects. Patients with an electrolyte imbalance are prone to poor prognosis after PCI, and the survival period without MACE within 90 days is significantly lower than that of normal patients.

## Figures and Tables

**Figure 1:** The relationship between electrolyte levels and the survival period of MACE in patients with acute STEMI.

**Table 1:** Comparison of general data of three groups of acute STEMI patients (*n*, mean ± SD).

General data	Normal group (*n* = 78)	Mild decline group (*n* = 46)	Severe decline group (*n* = 18)
Age (year)	52.45 ± 9.48	58.49 ± 11.28	65.12 ± 10.69
Gender (male/female)	40/38	25/21	9/9
History of diabetes (*n*, %)	17 (21.79%)	10 (21.74%)	5 (27.78%)
History of hypertension (*n*, %)	34 (43.59%)	19 (41.30%)	8 (44.44%)
Fasting blood glucose (mmol/L)	9.81 ± 2.15	10.24 ± 3.76	10.46 ± 4.12
Total cholesterol (mmol/L)	4.52 ± 0.68	4.63 ± 0.94	4.58 ± 0.72
Triglycerides (mmol/L)	1.52 ± 0.12	1.56 ± 0.14	1.48 ± 0.11
WBC (×10^9^/L)	9.77 ± 3.15	9.83 ± 3.21	9.94 ± 3.06
RBC (×10^12^/L)	4.68 ± 0.90	4.58 ± 0.88	4.63 ± 0.88
Hb (g/L)	137.88 ± 18.24	134.14 ± 17.29	138.64 ± 19.48
PLT (×10^9^/L)	215.07 ± 54.46	213.24 ± 51.75	211.08 ± 53.77
CK-MB (U/L)	103.45 ± 12.48	185.94 ± 20.67^*∗*^	269.73 ± 21.07^*∗*#^
CK (U/L)	2261.73 ± 220.61	2298.45 ± 256.37	3544.81 ± 247.19^*∗*#^
cTnI (*μ*g/L)	0.21 ± 0.08	1.26 ± 0.12^*∗*^	2.09 ± 0.11^*∗*#^
LVEF (%)	55.42 ± 4.65	48.43 ± 3.72^*∗*^	40.95 ± 4.08^*∗*#^
LVDP (mmHg)	74.49 ± 10.73	70.98 ± 11.68	72.44 ± 10.95
LVSP (mmHg)	125.67 ± 18.91	116.52 ± 15.99	117.58 ± 16.62
Myocardial infarction area (%)	13.90 ± 1.28	18.08 ± 1.41^*∗*^	22.04 ± 1.55^*∗*#^
Gensini score (points)	54.07 ± 10.14	62.18 ± 10.27^*∗*^	77.54 ± 11.51^*∗*#^

*Note*. Compared with the normal group, ^*∗*^*P* < 0.05. Compared with the mild decline group, ^#^*P* < 0.05.

**Table 2:** Analysis of multiple factors affecting electrolyte levels in patients with acute STEMI.

Influencing factors	*B*	*SE*	*Walds*	d*f*	Sig.	Exp (B)
CK-MB	1.558	0.428	7.192	1	0.032	4.236
CK	1.446	0.409	6.958	1	0.037	3.653
cTnI	1.975	0.473	9.075	1	0.008	6.072
LVEF	0.462	0.237	3.251	1	0.573	1.809
Myocardial infarction area	1.368	0.409	4.079	1	0.042	3.561
Gensini score	1.473	0.502	8.610	1	0.011	5.939

**Table 3:** Adverse conditions of three groups of acute STEMI patients within 90 days after PCI.

Group	*n*	Cardiogenic shock	Heart failure	Ventricular aneurysm	Ventricular septal perforation	Other events	Death
Normal group	78	5 (7.69%)	7 (8.97%)	1 (1.28%)	0 (0.00%)	2 (2.56%)	9 (11.54%)
Mild decline group	46	11 (23.91%)^*∗*^	8 (17.39%)^*∗*^	3 (6.52%)^*∗*^	1 (2.17%)^*∗*^	1 (2.17%)	13 (28.26%)^*∗*^
Severe decline group	18	6 (33.33%)^*∗*^	5 (27.78%)^*∗*#^	3 (16.67%)^*∗*#^	1 (5.56%)^*∗*#^	0 (0.00%)	10 (55.56%)^*∗*#^

*Note*. Compared with the normal group, ^*∗*^*P* < 0.05. Compared with the mild decline group, ^#^*P* < 0.05.

## Data Availability

The data used and/or analyzed during the current study are available from the corresponding author upon request.
